# Implementation of Combined Machine Learning with the Big Data Model in IoMT Systems for the Prediction of Network Resource Consumption and Improving the Data Delivery

**DOI:** 10.1155/2022/6510934

**Published:** 2022-07-19

**Authors:** M. Sugadev, Sonia Jenifer Rayen, J. Harirajkumar, R. Rathi, G. Anitha, S. Ramesh, Kiran Ramaswamy

**Affiliations:** ^1^Department of Electronics and Communication Engineering, Sathyabama Institute of Science and Technology, Chennai, Tamilnadu, India; ^2^Department of Information Technology, Jeppiaar Institute of Technology, Sriperumbudur, Chennai 631604, Tamil Nadu, India; ^3^Department of Electronics and Communication Engineering, Sona College of Technology, Salem 636005, Tamil Nadu, India; ^4^School of Information Technology and Engineering, Vellore Institute of Technology, Vellore 632014, Tamil Nadu, India; ^5^Department of Electronics and Communication Engineering, Saveetha School of Engineering, SIMATS, Chennai, Tamil Nadu, India; ^6^Department of Computer Science and Engineering, Saveetha School of Engineering, SIMATS, Chennai 602105, Tamil Nadu, India; ^7^Department of Electrical and Computer Engineering, Dambi Dollo University, Dembi Dolo, Ethiopia

## Abstract

In recent years, health applications based on the internet of medical things have exploded in popularity in smart cities (IoMT). Many real-time systems help both patients and professionals by allowing remote data access and appropriate responses. The major research problems include making timely medical judgments and efficiently managing massive data utilising IoT-based resources. Furthermore, in many proposed solutions, the dispersed nature of data processing openly raises the risk of information leakage and compromises network integrity. Medical sensors are burdened by such solutions, which reduce the stability of real-time transmission systems. As a result, this study provides a machine-learning approach with SDN-enabled security to forecast network resource usage and enhance sensor data delivery. With a low administration cost, the software define network (SDN) design allows the network to resist dangers among installed sensors. It provides an unsupervised machine learning approach that reduces IoT network communication overheads and uses dynamic measurements to anticipate link status and refines its tactics utilising SDN architecture. Finally, the SDN controller employs a security mechanism to efficiently regulate the consumption of IoT nodes while also protecting them against unidentified events. When the number of nodes and data production rate varies, the suggested approach enhances network speed. As a result, to organise the nodes in a cluster, the suggested model uses an iterative centroid technique. By balancing network demand via durable connections, the multihop transmission technique for routing IoT data improves speed while simultaneously lowering the energy hole problem.

## 1. Introduction

A person's health is essential for living a happy and successful life. Health is defined by the World Health Organization (WHO) as a state of physical and mental well-being that is devoid of illness or disability. Healthcare is the process of preventing, diagnosing, and treating illnesses and injuries in order to maintain or improve one's health. Traditional healthcare relies on manual management and maintenance of patient demographic data, case history, testing, prescriptions, billing, and drug stock maintenance, which leads to human errors and hurts patients. Smart healthcare based on the internet of things (IoT) reduces human mistakes by linking all critical parameter monitoring equipment over a network to a central computer. This helps physicians recognise illnesses more quickly and precisely. The internet of medical things (IoMT) refers to medical devices that may transport data across a network without requiring human-to-human or human-to-computer contact [1]. Gartner, a research and consultancy firm, predicts that by 2020, 20.4 billion devices will be connected to the Internet. Furthermore, by 2020, the worldwide IoT market will have grown at a 16.9% annual pace to 1.7 trillion dollars, up from 655.8 billion dollars in 2014. An IoMT platform is a smart system that includes sensors and electronic circuits for collecting biomedical signals from patients, a processing unit for processing the biomedical signals, a network device for transmitting biomedical data over a network, a temporary or permanent storage unit, and a data visualization platform for visualising the biomedical data. This substantial funding will also be utilised to develop IoMT systems [2].

The internet of things (IoT) is a paradigm shift that uses sensors and tangible objects to connect the physical and digital worlds. It works with a wide range of mobile devices and offers clever societal support options. Smart applications change the present system by distributing and ensuring the trustworthiness of academic and industrial data [3]. These systems are compatible with a wide range of wireless communication, portable device, and cloud computing components. The internet of medical things refers to wearable sensors that work with other medical equipment and clinical systems to aid in health-related activities (IoMT) [4]. They enable remote monitoring of a patient's condition, such as chronic illness management, blood pressure, and heartbeat. Modern health applications, on the other hand, greatly increase the volume of medical data that must be properly maintained, necessitating the use of big data analytics to analyse the data. While IoMT delivers a wide range of services to patients and the medical team, it also raises significant security and authentication challenges in terms of privacy concerns, particularly when dealing with sensitive medical data, according to various research studies [5].

Medical equipment and internet of things (IoT) technologies are combined in the internet of medical things (IoMT). With every medical gadget connected to the Internet and monitored by medical personnel, IoMTs are the future of healthcare systems. As technology advances, healthcare will be delivered faster and at a cheaper cost.  Figure 1 depicts an example of IoMTs in which patient vitals are acquired via sensor devices and transmitted via the Internet to IoMT apps. The data is passed on to healthcare professionals and medical personnel, who reply to the patient in question [6].

Machine learning approaches have recently gained prominence, and they use statistical analysis to learn from environmental data. This makes network applications smarter and prevents them from following a set of static rules [7]. With better network resource management and security assaults, the machine learning algorithm streamlines the decision-making process and improves performance for response time. Many systems use SDN architecture, which separates the control plane from the data plane to allow centralised control for effective network management. Furthermore, several methods for integrating SDN in the health business have lately been proposed because of the low-cost administration of IoT devices [8].

IoMT technologies have been widely adopted by various academics in recent years to enable efficient network systems. These technologies work in conjunction with a wireless network to collect data from patients' bodies and process it using advanced algorithms. Furthermore, the processed data is transferred to the sink node, where medical specialists can analyze it for disease diagnosis [9]. Medical devices, on the other hand, are severely limited in terms of numerous resources and are unable to perform high-cost data processing and storage. As a result, various solutions have been presented in the past to provide cloud-based services; nevertheless, it has been observed that certain systems are unable to protect sensitive data from threats [10]. Furthermore, due to their dynamic and heterogeneous character, typical security methodologies cannot be applied to limited constraint devices. However, few solutions have been presented for resolving security issues without adding to the overhead and administrative costs. In a wide variety of industries, lowering communication overheads and automating security policies using SDN is a difficult task. As a result, this study proposes a machine learning SDN-enabled big data model for IoMT systems that oversees optimal network resource management and optimises health data delivery [11]. Furthermore, employing SDN architecture lowers network management costs and lowers the overhead of the control plane over installed sensors. Furthermore, the SDN-enabled security mechanism effectively employs medical devices to secure sensitive data from security threats.

## 2. Related Work

### 2.1. Internet of Healthcare Things

The recent technology plays a growing role in the healthcare industry with the rise of eHealth and mHealth. Patients are implanted with millions of sensors that continually monitor their health based on physiological, environmental, and behavioural aspects. Wireless body sensor networks are a common tool for monitoring patients in healthcare IoT, such as eHealth and mHealth. Wireless body sensor networks have sensors all throughout the human body. Every layer has its own set of components and responsibilities. Wearable sensors and in-body sensors are among the sensing devices found in the sensing layer. Medical super sensors (MSS) are a new form of sensor node with increased memory, processing, and communication capabilities. Patients commonly wear or have these network-connected sensors implanted into their skin. For diabetes patients, these sensors capture crucial information such as body temperature, blood pressure, pulse rate, respiration rate, ECG, and blood glucose [12].

Actuators have been employed to raise warnings and adjust environmental factors as needed in recent years. The tremendous breakthroughs in these applications are witnessed in the form of innovative monitoring applications. As a result, these apps generate a massive amount of contextual data. When building devices at the sensor layer, big data, among other key issues, must be taken into account. Price, size, energy consumption, memory, processing, power, deployment, and organisation of diverse devices are all issues at this tier. The communication layer is analogous to the physical layer in the TCP/IP paradigm. This layer connects and distributes data among physical entities in the WBSN using specialised communication protocols. It makes communication across and within networks easier. WBSN interoperability is enabled through the standards and communication protocols developed at this layer. These protocols also make it easier to share data across existing infrastructures. At this layer, WSBN supports Bluetooth, ZigBee, RFID, NFC, and UWB, among other intercommunication technologies [13].

Network management and QoS (latency, congestion, and energy efficiency), as well as security and privacy, are all concerns. Data aggregation and big data analytics, on the other hand, should be researched further. The restricted processing capabilities of hardware components present a challenge at this layer. These methods help resource-constrained networks conserve energy by substantially reducing data transmission throughout the network. The third tier is the processing layer, which analyses the collected data, makes decisions, and sends out alerts and notifications. This layer's main components are the CPU unit, hardware platforms, and operating system. This layer's partially analysed data is subsequently delivered to the storage layer, which is the next layer. A vast number of devices may be linked to the human body in IoT healthcare, resulting in massive volumes of complicated data. The storage layer is responsible for effectively handling and storing such data in order to analyse and utilise it later. IoT-based systems are unable to store such data due to their limited memory [14].

ThingWorx, OpenIoT, Google Cloud, Amazon, Nimbits, and GENI are among the cloud-based data storage solutions available to address this issue. Data management and storage are aided by these technologies. Data may be accessed and seen from almost anywhere on the globe. This enables health practitioners and scholars to go further into the subject in order to have a better understanding and progress of the field. The mining and learning layer is in charge of big data analytics and knowledge extraction. Machine learning approaches for large data analytics have been successful in healthcare IoT. Machine learning-based solutions can handle massive datasets rapidly, learn from the data, and improve the learning experience. They are used to sift through large amounts of medical data to find important, perhaps exciting, and unique and hidden information [15].

### 2.2. Software Defined Network

The most promising future networking paradigm looks to be software-defined networking. The three levels of SDN are the application, control, and data planes, with north- and southbound APIs in between. Through network programmability, the SDN paradigm has broken down network administration to a vendor-independent architecture [16].

As the control plane and data plane have been split, SDNs have developed as a new networking paradigm. All control logic has been transferred to a centralised control plane because of SDN's novel and promising structure. The centralised design and intelligence of SDNs are the foundations of their strength and potential. An SDN controller uses the southbound protocol to gather information (statistics) from network devices. The southbound protocol, which is responsible for information transmission between the controller and networking devices, is the most important protocol in the SDN architecture. One of the most important southbound protocols is OpenFlow, a standard communication interface created by the Open Networking Foundation (ONF) and defined by an SDN architecture's data and control planes. This interface allows for direct access to and manipulation of the forwarding plane components of network devices such as routers and switches [17].

The SDN controller connects to the switch using the southbound API, with OpenFlow being the most used standard. Other options are NOS, RYU, and P4. Only a few examples are Floodlight, POX, and other open software for the NOS platform. The NOS's northbound API can be used to programme the network by SDN applications. The switch is linked to the controller, and the OpenFlow protocol is used to transport packets between the switch and the controller. The network, comprising all policies and actions, is under the authority of a controller [18].

There are legitimate concerns about SDN's scalability; nonetheless, scaling challenges are not exclusive to SDN. The design of a typical control protocol confronts the same challenges. As a result, rather than being concerned about SDN, we should be concerned about traditional network scaling issues. To maintain SDN's scalability, control applications should be built with the least amount of consistency possible. In a typical data centre, switching elements can grow quickly. The centralised controller cannot keep up with the quick rate of change in the network's control events. One way to avoid this problem is to install rules on the switches that remove control requests before they enter the system. The high volume of control channel traffic puts a strain on SDN, perhaps causing control messages to be delayed. Programmable network virtualization based on SDN is crucial in cloud architecture for accommodating a variety of services [19].

The internet of things generates a large amount of traffic; therefore, dynamic provisioning of virtual security services increases network edge scalability. SDN, on the other hand, is essential for network dynamic reconfiguration and instant delivery of new networking rules. SDN has shown to be a flexible and strong network solution enabler. Scalability, dynamism, adaptability, and centralised management are all advantages of SDN-based solutions, in addition to improved control decisions. The control plane of SDN is fully adjustable, allowing it to change a variety of functions. It can extend a number of networks on its data plane, including edge, fog, vehicular networks, and the internet of things [20].

## 3. Methodology

### 3.1. Architecture of IoMT

The IoMT architecture consists of things, fog, and cloud layers. The health-care experts can directly communicate with the user through the router and through the local processing server.  Figure 2 shows the architecture of IoMT with layers.

#### 3.1.1. Things Layer

The monitoring device, medical records, sensor, actuator, pharmacy control, and so on are consisted in the things layer [21]. The user of the ecosystem is directly connected to this layer. Patient monitoring data, data from wearable sensor, and remote care data are collected in this layer. The data used in this device are placed securely to ensure the collected data integrity [22]. These devices are connected to the fog layer that is responsible for the local router in the ecosystem [23]. The meaningful information is generated by preprocessing the data at the fog and cloud layers [24]. The experts in healthcare can get the data through the router to reduce the delay.

#### 3.1.2. Fog Layer

This layer operates between the cloud and things layers, which consist of a server and gateway device for distributed network framework. For real-time users, the lower layer device is get harnessed the local processing power. This serves as the users to manage the security and integrity of the proposed IoMT system [25]. The data are redirected from the server to the cloud layer. The expert can get the data of the patient through the router to reduce the delay.

#### 3.1.3. Cloud Layer

The data storage and the resource computation for the data are analysed in this layer. The decision-making system is derived based on resource computation [26]. A huge medical data is incorporated into the cloud, and the operation of the healthcare system is handled easily. The data generated from the cloud resource is stored and analysed using the medical infrastructure.

### 3.2. SDN in IoMT

The IoMT is divided into two parts in the network: data plane and control plane [27]. The traffic is forward towards the destination from data plane, and the necessary task is performed using the control plane that allows forwarding decisions. A standard way to communicate the data and control plane is provided by software-defined networking (SDN)

The interface between the data and control plane used standard SDN protocol to make the system standard. The data plane is collected from the external server with a lot of different data using the standard open flow protocol. This makes the development of healthcare applications [28]. The proposed SDN-enabled IoMT is shown in Figure 3. The healthcare application is connected to the IoMT device in which the cloud is located through the control plane of SDN [29]. The data from IoMT are collected in the control plane of SDN, and the healthcare application is provided that has the privacy and security application where the diagnosis of patient or safety application is provided.

### 3.3. Proposed SDN Model

The proposed model is given in this section. The proposed system consists of machine learning and software-defined network algorithms. The main component in the proposed system is given in Figure 4.

Sensors, actuators, and communication devices make up the sensing layer, which collects data from patients and interacts with them to complete the transmission system. SDN routers, switches, and controllers are used in the second layer to manage IoT resources more efficiently by improving their performance in terms of computing power and energy usage. Furthermore, rather than direct communication between IoT nodes and the application layer, the suggested approach makes use of the SDN controller's intelligent capabilities and uses a controlled flooding method to avoid wasting resources [30].

The application layer houses the e-health services that work with IoT data to help the medical team diagnose a sickness or illness and treat it appropriately. The SDN controller reduces the overheads on restricted resources for IoT devices while guaranteeing data privacy and centralised management by employing a security strategy [31]. As a result, all of the layers work together to improve the performance of IoMT systems in a smart and secure way. The control plane in the proposed approach is meant to use centralised administration for data routing and security procedures. It was in charge of the data plane, which was responsible for maintaining the forwarding tables.

There are two algorithms in the proposed model. The first is for identifying IoT nodes using machine learning and reducing connection distance while lowering administration costs. It also decreases computational overloads on the channels and eliminates superfluous data redirection. The second method makes use of the SDN controller's customizable structure to create a centralised security system. The controller maintains track of the IoT layer's global data and efficiently controls the node's resources. It provides high-level security for an unpredictably changing environment by safeguarding critical data against attacks and managing network resources intelligently.

It provides high-level security for an unpredictably changing environment by safeguarding critical data against attacks and managing network resources intelligently. To begin, the suggested approach uses mean shift clustering, an unsupervised machine learning technique that groups IoT sensors into different collections. The proposed model, unlike most other current methodologies, does not take into account predefined network constraints.

The neighbour node is slightly moved to the transmission radius. The mean for the node as the enclose sensor position is given as follows:

(1) $$\begin{array}{c} M_{s}=\sum_{i=1}^{N}Y\times \left[\frac{\left(x_{i}-x\right)x_{i}}{x_{i}-x}\right], \end{array}$$

where *Y* is the number of iterations.

The neighbours are updated in each cycle using the source node's transmission radius. As a result, the suggested approach iteratively groups each IoT sensor to the cluster's nearest centroid point. Following that, the distance and connection estimate factors are used to pick cluster heads. Each cluster head is exclusively associated with specific nodes and serves as an edge manager. The selection of cluster method *f* is given as follows:

(2) $$\begin{array}{c} f\left(a\right)=\text{min}\left(d\left(a\right)\times \text{max}\left(l\right.\left(a\right)\right), \end{array}$$

where *d*(*a*) is distance of node form the centroids, 1(*a*) is performance measurement of link, and *f*(*a*) is cluster head selection.

The control plane and data plane are separated in SDN, and the controller has a global view of the complete network topology. The control plane in the proposed model keeps track of network entries, which include node statistics, wireless channel priority, and route information. On specific occurrences, the stored entries are dynamically updated. The control plane is created and programmed to decide how routes are picked for network routing and support an intelligent decision-making system using this information. The controller effectively retrieves the stored data and makes the best use of network resources in terms of energy efficiency, communication bandwidth, and load sharing. Later, the data plane employs network devices and sensors to carry out data flow in accordance with the control plane's regulations. The condition of links is determined using the statistic of node and maintaining the process of forwarding. The computation of resources is dependent on the performance metrics such as latency, reception rate, and time interval for packet. The proposed model is trained under SDN control using updated values of such realistic metrics to forecast efficient connections as a source of routing. In addition, at the end of the predetermined period, the most recent data are sent to the control plane, bringing the network records up to date.

The data plane is separated from the control plane using the SDN, and the entire structure of the network is controlled by the global view of the controller. The network entries are maintained by the control plane in the proposed system, which consists of route information, statistics of nodes, and the wireless channel priority.

The control plane is analysed using the information based on the entities that are stored and updated dynamically and decided by programming the routes, and network routing is achieved, and decision-making is carried out in the system using the intelligent support. The stored information is obtained efficiently using the controller, and the network resource is exploited based on load sharing, bandwidth communication, and efficient energy. The rules implanted are based on the flow of sensor that utilized the data plane for the network device to accomplish the flow of data. The condition for the link is determined using the statistics of a node using the function status *s*(*n*), and the forwarding process is accomplished. The computation of state function *s*(*n*) depends on the round-trip latency *L*_*rt*_(*n*), which is a realistic metric, and the reception rate of packet *P*_*rr*_(*n*) in a time interval *T*. The computation function is given as follows:

(3) $$\begin{array}{c} s\left(n\right)=\min\left(L_{rt}\left(n\right)+\max\left(P_{rr}\left(n\right)\right)\right). \end{array}$$

Under the control of SDN, the value of realistic metrics is updated, in which the proposed model is trained to determine the effective link for routing of source. The control plane gets the latest information at the end of the present interval to make the record of the network update.

The round-trip latency is minimum with a high reception ratio of packets considered according to the suitable link. The data from the IoT move to the SDN layer, which comprises router, controller, and switches. The open flow protocol is used to maintain communication among the central controller and switches. The role of the gateway is performed using the switches that offer the service of dual-level opportunities and manage the communication based on the trust orientation with the controller in the centralised system. The data in the network is secured again the IoT network threat. The security algorithm with high cost is executed using the SDN controller, and the power of gateway and nodes in IoT is lowered.

The trust certificates are generated using the SDN controller and in an authentic manner and securely. Reliable communication is offered by the trusted certifies which avoids the flooding of traffic in malicious and packet distribution. The trusted certificate has data and signatures for a particular gateway node. The data plane consists of ID and key associated with the RSA algorithm. The digital signature comprises the signature part with a centralized controller with the private key. The trusted certificate obtained from the gateway of the controller is given as follows:

(4) $$\begin{array}{c} C_{r}⟶T_{cer_{a}}=E\_P_{r}\left(ID_{a},k_{a}\right),\\ C_{r}⟶T_{cer_{b}}=E\_P_{r}\left(ID_{b},k_{b}\right). \end{array}$$

The trusted certificate is received by interchanging the nodes of the gateway and maintaining authentication and becoming the network service. The public key generated is distributed and maintains validity and authenticity and securely stores the threats anonymously. The function randomized encryption *E* for IoT layer with data in node *d*_*i*_; encrypted utilizing *r*_*i*_ is given as follows:

(5) $$\begin{array}{c} E:C_{i}=d_{i}\times k_{i}\left(r_{i}\right)+v_{i}. \end{array}$$

Figure 5 depicts the working flowchart of the proposed model. Until IoT nodes are sorted into collections, data from IoT networks and repeat-generated centroids using neighbours are the two main components. After that, near-optimal pathways from the IoT network layer to SDN switches are predicted without making any assumptions. The SDN component of the proposed approach manages network resources and load balance of the IoT network. The SDN gateways operate with the centralised controller to implement security against malicious and unauthenticated nodes. It monitors network activity using trustworthy certificates and begins the routing process in a systematic manner. When the recommended model receives a request for assistance from an application user, it first verifies their credentials, and if they are accepted, the cloud servers offer the desired service. If a malicious request node is found, its identification is identified as wrong, and inbound requests are refused. Furthermore, signed keys are generated between cloud servers and application users in order to generate encrypted blocks and ensure privacy through authentication.

## 4. Result and Discussion

The proposed technique improves network speed when the number of nodes and data generation rate fluctuate. As a result, the proposed model employs an iterative centroid approach to arrange the nodes in a cluster. Furthermore, each cluster has a cluster head who is more efficient than the other nodes. The multihop transmission approach for routing IoT data enhances speed while also reducing the energy hole problem by balancing network demand via durable connections. When the number of nodes and data production rate varies, the suggested approach enhances network speed. As a result, to organise the nodes in a cluster, the suggested model uses an iterative centroid technique. Each cluster also has a cluster leader, who is more efficient than the other nodes. By balancing network demand via durable connections, the multihop transmission technique for routing IoT data improves speed while simultaneously lowering the energy hole problem.  Figure 6 shows the throughput performance.

Due to the implementation of a machine learning technique to assist the nodes in forwarding data packets with minimal congestion and realistic parameters based on the cooperative work of SDN switches and controllers, the suggested model improves the packet loss ratio. Malicious entries are also flagged as faulty for future communications, and unknown nodes are not permitted to join the routing system. The SDN layer gateways not only provide security for the IoT network but also make it easier for the controller to update the network's global knowledge. This type of technology makes it easier to spot broken links and makes greater use of transmission capacity. In addition, the number of unauthenticated connections to the IoT network is reduced, and data are safely delivered to cloud servers via secured paths. Unlike prior solutions, the proposed model uses SDN architecture to efficiently use restricted resources and smoothly handle node data delivery.  Figure 7 shows the packet drops ratio performance.

In terms of faulty data packets, the confirmed outcome of the suggested model is depicted in Figure 8. The suggested methodology improves the ratio of defective data packets. The centralised controller and SDN gateway are in charge of establishing trust and maintaining data security among constrained nodes in the proposed approach. The centralised administration of SDN not only decreases the burden on the IoT network but also handles the privacy and authentication for specified routes. As a result, in IoT networks, only trustee nodes are permitted to submit and receive route requests over the fault-tolerant link. Furthermore, trustworthy nodes securely share their key information for data encryption and integrity, ensuring that only legitimate users have access to data. Furthermore, cloud servers and application users generate signed secret keys, which aid in the timely identification of rogue users and provide a low-cost data security technique. Such an algorithm rejects malicious node requests and marks them as defective, preventing further requests from the same identity from being processed.

Figure 9 compares the suggested model's performance in terms of data latency. It is found that it efficiently and timely enhances the network data ratio. It takes into account congestion levels to forecast the best channels for transferring data from the IoT layer to the cloud layer, all while being managed by the SDN controller. Furthermore, the SDN design enables constraint-oriented nodes to reduce their battery use and transfer data more quickly with a longer route duration. Furthermore, the network performance prevents frequent network disconnectivity owing to the balance of energy, link, and transmission load in routing between formed clusters. The suggested approach makes effective use of SDN's resilient architecture by utilising gateways and updating connection information on the controller. The proposed model reduces the unacceptably long time it takes for data to arrive. Furthermore, trustworthy certificates identify fraudulent nodes in a timely manner, preventing defective nodes from dropping actual data, resulting in a considerable reduction in transmission latency.

Figure 10 compares the proposed model's confirmed outcome for the use of energy resources with and without an SDN controller. The experimental findings show that the scenario with SDN deployment effectively exploits energy efficiency while lowering consumption. Experiments are carried out using a variety of nodes and data production rates. The suggested approach is based on SDN technology and the OpenFlow protocol, which allows for centralised network infrastructure management. The controller in the proposed model uses passive monitoring to monitor data plane entities and updates the information of wireless channels with valid route entries.

As a result, the SDN controller dynamically manages the constraint nodes and gateways based on network circumstances. Using the knowledge gained from the lower layer explicitly reduces overheads and increases energy efficiency. Furthermore, the programmed control plane expressly employs the set of criteria and selects forwarder nodes to balance the burden of energy consumption. Furthermore, for effective bandwidth and resource management, the controller retrieves the stored information from the data plane. However, because there is no global database on the central point and each node communicates with others using its resources, the scenario without SDN wasted too much energy in various operations. Furthermore, due to the lack of a centralised controller, the majority of sensor data is lost or even retransmitted, consuming extra network resources.

## 5. Conclusion

This paper identified a machine-learning approach with SDN-enabled security for reducing network usage and ensuring timely delivery of IoT services. Over the deployed IoT network, the SDN centralised architecture is employed to eliminate the control plane overhead. It groups the nodes using machine learning iterative centroid computation and enhances routing efficiency in a realistic setting. The created routing strategy is used in conjunction with the SDN controller to provide a secure chain with minimal overheads and energy consumption. Furthermore, the overload links are not used in routing decisions when evaluating the status function. In the future work, the overload link will be considered in the routing decision.

## Figures and Tables

**Figure 1:** Basic architecture of IoMT.

**Figure 2:** Architecture of IoMT with layers.

**Figure 3:** IoMT enabled with SDN.

**Figure 4:** Proposed SDN system.

**Figure 5:** Flow diagram of proposed SDN system.

**Figure 6:** Throughput performance: (a) based on the number of nodes and (b) rate of packet generation.

**Figure 7:** Packet drops ratio performance: (a) based on the number of nodes and (b) rate of packet generation.

**Figure 8:** Performance of packet with fault: (a) based on the number of nodes and (b) rate of packet generation.

**Figure 9:** Data delay performance: (a) based on the number of nodes and (b) rate of packet generation.

**Figure 10:** Energy consumption of the network: (a) based on the number of nodes and (b) rate of packet generation.

## Data Availability

The data used to support the findings of this study are included within the article and further data or information can be obtained from the corresponding author upon request.

## References

[1] Ud Din I., Almogren A., Guizani M., Zuair M. (2019). A decade of internet of things: analysis in the light of healthcare applications. *IEEE Access*.

[2] Chai W., Khan Y., Jan F. (2021). Comprehensive survey on machine learning-based big data analytics for IoT-enabled smart healthcare system. *Mobile Networks and Applications*.

[3] GatouillatGatouillat A., Badr Y., Massot B., Sejdic E. (2018). Internet of medical things: a review of recent contributions dealing with cyber-physical systems in medicine. *IEEE Internet of Things Journal*.

[4] Hayajneh A. A. I., Bhuiyan M. Z. A., McAndrew I. (2020). Improving internet of things (IoT) security with software-defined networking (SDN). *Computers*.

[5] Janke A. T., Overbeek D. L., Kocher K. E., Levy P. D. (2016). Exploring the potential of predictive analytics and big data in emergency care. *Annals of Emergency Medicine*.

[6] Vishnu S., Ramson S. R. J., Jegan R. Internet of medical things (IoMT) - an overview.

[7] Koutras D., Stergiopoulos G., Dasaklis T., Kotzanikolaou P., Glynos D., Douligeris C. (2020). Security in IoMT communications: a survey. *Sensors*.

[8] Sendrayaperumal A., Mahapatra S., Parida S. (2021). Energy auditing for efficient planning and implementation in commercial and residential buildings. *Advances in Civil Engineering*.

[9] Gopalan A., Kommuri U. K. (2018). Design and development of miniaturized low voltage triangular RF MEMS switch for phased array application. *Applied Surface Science*.

[10] Jain D. K., Tyagi S. K. S., Neelakandan S., Prakash M., Natrayan L. (2022). Metaheuristic optimization-based resource allocation technique for cybertwin-driven 6G on IoE environment. *IEEE Transactions on Industrial Informatics*.

[11] Mukhtar H., Rubaiee S., Krichen M., Alroobaea R. (2021). An IoT framework for screening of COVID-19 using real-time data from wearable sensors. *International Journal of Environmental Research and Public Health*.

[12] Kaur P., Sharma M., Mittal M. (2018). Big data and machine learning based secure healthcare framework. *Procedia Computer Science*.

[13] Fu H., Mohamed C., Al Ali A. (2020). Multi-layer security scheme for implantable medical devices. *Neural Computing & Applications*.

[14] Vaishali K. R., Rammohan S. R., Natrayan L., Usha D., Niveditha V. R. (2021). Guided container selection for data streaming through neural learning in cloud. *International Journal of System Assurance Engineering and Management*.

[15] Rajagopalan K., Angalaeswari A., Natrayan S., Mammo L., Mammo W. D. (2022). Combined economic emission dispatch of microgrid with the incorporation of renewable energy sources using improved mayfly optimization algorithm. *Computational Intelligence and Neuroscience*.

[16] Ramasubramanian B., Anitha G. (2012). An efficient approach for the detection of new vessels in diabetic retinopathy images. *Int. J. Eng. Innov. Technol*.

[17] Nehra S., Kumar M., Dilbaghi R. (2021). Internet of medical things (IoMT)-integrated biosensors for point-of-care testing of infectious diseases. *Biosensors and Bioelectronics*.

[18] Javeed D., Gao T., Khan M. T. (2021). SDN-enabled hybrid DL-driven framework for the detection of emerging cyber threats in IoT. *Electronics*.

[19] Asha P., Natrayan L., Geetha B. T. (2022). IoT enabled environmental toxicology for air pollution monitoring using AI techniques. *Environmental Research*.

[20] Sundaram S. S., .Hari Basker N, Natrayan L. (2019). Smart clothes with bio-sensors for ECG monitoring. *International Journal of Innovative Technology and Exploring Engineering*.

[21] Anupama C. S. S., Natrayan L., Laxmi Lidia E. (2021). Deep learning with backtracking search optimization-based skin lesion diagnosis model. *Computers, Materials & Continua*.

[22] Razdan S., Sharma S. (2021). Internet of medical things (IoMT): overview, emerging technologies, and case studies. *IETE Technical Review*.

[23] Syed L., Jabeen S., Manimala S., Alsaeedi A. (2019). Smart healthcare framework for ambient assisted living using IoMT and big data analytics techniques. *Future Generation Computer Systems*.

[24] Kumar R., Tripathi R. (2021). Towards design and implementation of security and privacy framework for internet of medical things (iomt) by leveraging blockchain and ipfs technology. *The Journal of Supercomputing*.

[25] Liaqat S., Akhunzada A., Shaikh F. S., Giannetsos A., Jan M. A. (2020). SDN orchestration to combat evolving cyber threats in Internet of Medical Things (IoMT). *Computer Communications*.

[26] Magesh S., Nivetha V. R., Rajakumar P. S., Radha RamMohan S., Natrayan L. (2020). Pervasive computing in the context of COVID-19 prediction with AI-based algorithms. *International Journal of Pervasive Computing and Communications*.

[27] Kanimozhi G., Natrayan L., Angalaeswari S., Paramasivam P. (2022). An effective charger for plug-in hybrid electric vehicles (PHEV) with an enhanced PFC rectifier and ZVS-ZCS DC/DC high-frequency converter. *Journal of Advanced Transportation*.

[28] Sahoo K. S., Puthal D. (2021). SDN-assisted DDoS defense framework for the internet of multimedia things. *ACM Transactions on Multimedia Computing, Communications, and Applications*.

[29] Montazerolghaem A. (2022). Defined internet of multimedia things: software-defined internet of multimedia things: energy-efficient and load-balanced resource management. *IEEE Internet of Things Journal*.

[30] Cecil J., Gupta A., Pirela-Cruz M., Ramanathan P. (2018). An IoMT based cyber training framework for orthopedic surgery using Next Generation Internet technologies. *Informatics in Medicine Unlocked*.

[31] Perwej Y., Ahamad F., Khan M., Akhtar N. (2021). An empirical study on the current state of internet of multimedia things (IoMT). *IJERCSE*.

